This article has been retracted.

# Optimal Allocation of Enterprise Resources Based on the Intelligent Algorithm from the Perspective of Multidimensional Dynamic Innovation

**DOI:** 10.1155/2022/1426201

**Published:** 2022-10-10

**Authors:** Wei Song, Zi Lin

**Affiliations:** Nanjing Audit University Jinshen College, Nanjing 210000, Jiangsu, China

## Abstract

Faced with the upsurge of digital technology, many small and medium-sized startups are aware of the opportunities and challenges it brings and are actively responding to digital transformation. Digital transformation is a type of strategic change with certain risks. On the one hand, this requires business leaders to have a sense of change, and on the other hand, it also requires certain resources to be invested. As a result, in the real world, not all small and medium-sized entrepreneurial firms have the ability or inclination to implement digital transformation. SMEs' digital transformation has become a key factor in promoting the national economy's transition from new and old kinetic energy and providing new prospects for development of small and medium firms. As a starting point, this study devises an index system for assessing the digital maturity of small and medium-sized businesses. Based on the AHP method in the multicriteria framework, a hierarchical structure is established for each index, a three-layer basic framework is established, and the weight of the evaluation index is calculated. Second, this work establishes a BP network model for digital transformation maturity assessment of startups based on AHP and establishes a three-layer BP network structure. This work aims to optimize BP network using the improved ISFLA algorithm. It improves the adaptive step size update formula in the SFLA algorithm by using the mutation operator and improves the evolution method of the worst individual of the frog to the simultaneous evolution of multiple poor individuals. The constructed ISFLA-BP algorithm is then used to evaluate the digital transformation maturity of small and medium-sized startups. Finally, systematic and comprehensive experiments are carried out to verify superiority as well as feasibility of the method.

## 1. Introduction

Entering the 2020s, the digital economy has become a major trend in enterprise development. On the one hand, the communication infrastructure represented by 5G is developing rapidly, network chips and smartphones have become popular, and social interconnection and the Internet of Everything have become a reality. On the other hand, technologies such as cloud computing, machine learning, and artificial intelligence have begun to emerge, which can conduct real-time dynamic analysis based on big data and better help entrepreneurs make scientific decisions. Today's world is in an era of great change in transition from an industrial economy based on resources and knowledge to a digital economy based on networking and data. Additionally, the digital economy serves as a catalyst for the movement of new and old kinetic energy in the economy, as well as an opportunity for businesses to change lanes and overtake. As a whole, the national strategy seeks to drive production techniques through digital transformation and to empower the transformation and upgrading of traditional industries. For small and medium-sized businesses, digital transformation is no longer an option, and it is a requirement for survival and long-term growth [1–7].

In the face of the ups and downs of digital technology, many companies are aware of the opportunities and challenges they bring and actively respond to them. The first level is to realize digitalization in a specific activity of the value chain and actively adopt digital technology in functional activities such as engineering, marketing, supply chain, and financial management to improve departmental efficiency. Many companies now introduce digital marketing, business-finance integration systems, digital R&D platforms, and more. The second level is to digitize the products and services provided and improve the intelligence of the products, and use the APP, the Internet, and social platforms to connect with users to achieve seamless connection between products and customers. Many traditional manufacturing companies install sensors and chips on their products and connect them to mobile phones through software so that customers can manage smart products through mobile phones. The third level is strategic transformation or business model reengineering based on digitalization. Now some clothing companies are moving from traditional mass production to mass private customization based on individual needs of customers. The fourth level is to transform the entire industry ecosystem by introducing digitization. The traditional offline training and education industry has turned to online during the epidemic period, and the entire education industry is undergoing earth-shaking changes [8–16].

The digital economy's growth is being fueled by digital transformation. The digital transformation of small and medium-sized entrepreneurial firms is significant in the next phase of global industrial transformation through the integration and invention of digital technology and traditional inventive organizations. Small and medium-sized enterprises are focal point and key to strengthening supply-side structural reform, fostering high-quality development of businesses, and further growing the digital economy as a whole, as digital technology is increasingly applied at scale. Entrepreneurial small and medium-sized businesses are the pillars of the national economy and the source of power for economic growth. SME digital transformation has shifted the focus of national development from small to medium-sized firms. As compared to the world's most industrialized nations, they nonetheless face a wide range of challenges. As a result of a decline in factor endowment advantages, an imbalanced industrial structure, lack of core competitiveness, and insufficient autonomous innovation ability, an immediate action is required. To achieve high-quality development and empower small and medium-sized businesses to restructure and modernize, the government made it plain that digital technology was required. Entrepreneurial small and medium-sized businesses, as the main and cornerstone of the national economy, must achieve effective digital transformation and upgrading as quickly as possible. New and old kinetic energy can be transformed into high-quality development by completing a digital transformation of firms under digital technology's leadership, as well as by intelligently updating existing enterprises [17–19].

Evaluation for enterprises' digital transformation maturity is significant in digital transformation process. First, this work establishes an evaluation index system for the maturity of digital transformation of small and medium-sized entrepreneurial enterprises, establishes a hierarchical structure for each index via the AHP method in the multicriteria framework, establishes a three-level basic framework and calculates the weights of evaluation indicators. Second, this work establishes a BP network model for enterprise digital transformation maturity assessment based on AHP and establishes a three-layer BP network. This work aims to optimize BP network using the improved ISFLA algorithm. It improves the adaptive step size update formula in the SFLA algorithm by using the mutation operator and improves the evolution method of the worst individual of the frog to the simultaneous evolution of multiple poor individuals. The constructed ISFLA-BP algorithm is then used to evaluate the digital transformation maturity of small and medium-sized startups. Finally, systematic and comprehensive experiments are carried out to verify the superiority and feasibility.

## 2. Related Work

Literature [20] explains that digital economy provides impetus and technical support for the transformation and upgrading of enterprises. Digital transformation could promote the economic benefits of digital transformation of physical enterprises by reducing the cost of enterprises, improving efficiency for asset use, and enhancing innovation capabilities. Literature [21] discussed the benefits that digital transformation of enterprises could bring to enterprises from an economic perspective, which explained the fundamental reasons for enterprises' cross-system transformation. This could bring certain enlightenment to enterprises in the actual transformation and integration process. Literature [22] studied the digital transformation for enterprises and firstly expounded the inevitable trend for digital transformation of enterprises and then put forward suggestions to promote the information transformation of manufacturing enterprises, providing reference and experience for manufacturing enterprises to carry out digital transformation. Literature [23] believed that in the era of intelligence, enterprises should not only improve their cognition in terms of ideas and concepts, but more importantly, they should create a new capability system and realize the transformation of the enterprise by means of the change of the capability system itself. For the first time, it proposed a traditional enterprise transformation capability system that combined six key capability elements to provide reference guidance for digital transformation of enterprises. According to literature [24], a four-in-one support system should be built for the digital economy to foster the development of high-quality firms. The key to assisting businesses in their digital transformation was interpreted from four different angles in this document. The digital transformation of small and medium-sized organizations in digital economy age was examined in literature [25] by looking at some of the obstacles that small and medium-sized businesses face in their development. Studies in Refs. [26, 27] analyzed to identify common challenges, drivers, and opportunities for enterprise transformation. It provided a systematic overview of the digital transformation of enterprises by covering the technical, strategic, managerial, and organizational perspectives of the digitalization of the manufacturing industry, integrating insights from multisectoral and multidimensional analysis. The transformation and upgrading of enterprises in developed regions were not limited to digitalization, and relevant experts and scholars had proposed ideas and methods for the transformation to FOF.

Literature [28, 29] believed that the outbreak of the epidemic had forced small and medium-sized enterprises to carry out digital transformation. In order to resume work and production as soon as possible, many enterprises used online office platforms for online office, information sharing, and online learning and training. Reference [30] studied the digital transformation of a specific operation sector of an enterprise and discussed the motivations of digital transformation from the perspective of overall efficiency and data value. It is believed that there are three major driving forces: one was to achieve the connection between various links within the enterprise, and the requirements for data sharing with customers, suppliers, and fund providers; the second was to improve efficiency, reduce manpower consumption, and make better use of human resources; the third was to build data resources and conduct big data analysis to provide support for management decisions. Reference [31] defined digital transformation as a combination according to the four attributes of target entity, scope, method, and expected result. These triggers significantly changed entity properties, thereby improving the entity's process. Digital technologies caused disruption in the process, thus triggering a strategic response from organizations seeking to change the path to value creation. Enterprise digital transformation was characterized as an organizational shift to big data, analytics, cloud, mobile, and social media platforms [32]. To keep up with the ever-changing business environment, organizations must undergo digital transformation, which relied on new digital technologies to bring about distinctive changes in corporate operations, procedures, and the production of new value. According to literature [33], digital transformation of enterprises usually involved three stages: clarifying the mode of digital transformation, utilizing digital technology and customer needs to carry out comprehensive digital transformation, and changing the overall organizational model of the enterprise. Digital transformation, according to literature [34], could be defined as an enterprise's innovation process that incorporates both technological and strategic aspects. Organizational structure, procedures, competencies, and culture were needed to be reshaped to adapt to the rapidly changing digital world. Literature [35] believed that the digital transformation of enterprises was not just a construction at the technical level but required the use of digital technology to completely optimize and change organizational structures and processes. The key to transformation was laid in the adaptation of enterprises to changes in the market environment and changes in their cognitive models.

## 3. Method

First, this work establishes an evaluation index system for the maturity of digital transformation for small and medium-sized entrepreneurial enterprises, establishes a hierarchical structure for each index via the AHP method in the multicriteria framework, establishes a three-level basic framework, and calculates the weights of evaluation indicators. Second, this work establishes a BP network model for enterprise digital transformation maturity assessment based on AHP and establishes a three-layer BP network. This work aims to optimize BP network using the improved ISFLA algorithm. It improves the adaptive step size update formula in the SFLA algorithm by using the mutation operator and improves the evolution method of the worst individual of the frog to the simultaneous evolution of multiple poor individuals. The constructed ISFLA-BP algorithm is then used to evaluate the digital transformation maturity of small and medium-sized startups.

### 3.1. Evaluation Index System Construction Based on AHP

To build a relatively scientific, reasonable, and comprehensive evaluation index system for digital transformation maturity, certain principles need to be followed when designing the index system. The following principles must be observed when selecting and determining the digital transformation maturity evaluation indicators of small and medium entrepreneurial enterprises. The first principle is the principle of completeness. Small and medium-sized businesses' digital transformation maturity must be assessed from many angles and views, and an index system must be developed to measure this. In order to assess how well small and medium-sized businesses are preparing for the digital revolution, this system is used. The second is the principle of significance. The more comprehensive the evaluation indicators are selected, the better. Too many indicators will cause the indicators to fold and cross each other. On the other hand, the information obtained from the evaluation data is large, and the selected indicators should be targeted and representative to reflect the entire maturity evaluation effect in a timely manner. This is the goal of the examination of small and medium-sized organizations' digital transformation maturity. The operational principle is the third. Qualitative and quantitative indicators make up the comprehensive evaluation index system, and the qualitative indications must be quantified. All indicators can be assigned and measurable, and the data of evaluation indicators can be collected; otherwise, the setting of the indicators has no meaning. The digital transformation maturity evaluation index system of small and medium-sized entrepreneurial enterprises designed includes four dimensions, and each dimension contains more detailed divisions.

The first is strategy, where strategic metrics are primarily used to capture the maturity of an enterprise's digital strategy. Digital transformation awareness must be rooted in strategy, and the corporate strategy should be tested from a digital perspective, including the overall strategy and part of the strategy of each business unit. The achievement of modern business goals requires an information systems strategy process that is implemented in a continuous, dynamic manner between information technology and business. The management of the company must formulate a development strategy. The complete strategy includes development planning, special planning, and planning implementation.

The second is management. The management that is involved in the process of enterprise digital transformation is digital management, which refers to use of digital technology to informatize as well as automate front-end business processes such as R&D, procurement, production, and sales and to improve enterprise production efficiency. To measure digital management maturity of small and medium-sized startups, it is necessary to analyze the production management, quality management, design management, R&D management, order management, and procurement management of the enterprise.

The third is technology application. The application of new technologies is a basic requirement for digital transformation. First of all, digital transformation requires technology. Technology is the most important factor affecting the level for digitalization, and it is also the main focus of traditional digital technology upgrades. As the core element of digital transformation, technology should not be underestimated, and enterprises need to strengthen the upgrading and emphasis on new technologies. Secondly, at the technical level, the weight of digital investment and digital R&D capability indicators is relatively large, reflecting that digital investment is significant in transformation and development. Finally, the application of digital technology is the foundation of innovation; therefore, IT departments and business departments of enterprises need to cooperate more closely on digital transformation, strengthening the business capabilities within IT and the IT knowledge of executives. The selected subindicators are digital input, digital R&D, digital application, and digital output.

The fourth is the organizational structure. Digital transformation has brought important changes to the organizational structure of enterprises and improved the operational efficiency of enterprises. The higher the corporate status of the leader of the digitalization sector, the more obvious the advancement of digitalization. The number of enterprise management levels can reflect the organizational structure model of the enterprise. The fewer the number of enterprise management levels, the more flattened the enterprise organizational structure is. This can quickly adapt to the uncertainty brought about by technological change and improve the overall efficiency of the organization. As consumer demands become increasingly personalized, companies must use digital technology to transform their organizational structures to increase their responsiveness to the market. How to build a flat organizational structure to improve the overall efficiency of organization is a challenge faced by enterprises in the process of digital transformation. The selected subindicators include management levels, management departments, and digital department leadership. The evaluation index system of digital transformation maturity is demonstrated in Figure 1.

Weighting the evaluation indicators for small and medium-sized entrepreneurial companies' digital transformation maturity is a crucial step as the weight is used to measure the value that each index has in relation to reaching a specific goal. The value of quantitative and qualitative indicators for the evaluation of the maturity of digital transformation of small and medium-sized entrepreneurial firms must be converted into a comprehensive value using particular methodologies and regulations. Alternatively, you can reduce the multicriteria decision-making problem to a single-objective decision-making problem and then establish the index weight of the assessment system. In the evaluation process, the index weight reflects the different importance aspects of each index. Reasonable distribution of the weight is very important to the evaluation result. If the weight of an evaluation index changes, it will also have a great impact on the entire target evaluation result. Therefore, the setting of weights for the evaluation indicators of digital transformation maturity for small and medium entrepreneurial enterprises must be objective and scientific.

It is possible to integrate quantitative index analysis with qualitative index analysis when using AHP, which is a decision-making process with several criteria and objectives. AHP is based on the premise that a goal can be broken down into smaller goals based on the nature of the problem and the desired outcome. The elements are aggregated and merged at various levels according to the varying influences among the factors, resulting in an analytical structure model with many levels. Finally, the issue is on determining the relative important weights of the bottom layer and the ordering of relative superiority and inferiority.

Building a hierarchical structure, creating a judgment matrix, single-order and one-time inspection of hierarchical elements, and the total order of hierarchical elements and one-time inspection are the four processes in the AHP model construction process. A hierarchical model is important when employing AHP to tackle decision analysis problems. The target, criterion, and scheme layers make up the three main divisions of the hierarchical model. The construction of judgment matrix starts from the middle layer of the hierarchical model, that is, the element layer. The factors at this level are compared with each other, and the importance of the qualitative results can be calculated from the quantitative results so that a judgment matrix can be constructed. Specific quantitative methods are demonstrated in Table 1. Then construct a judgment matrix according to the values obtained in the table.

The largest eigenvalue and the corresponding eigenvector are obtained by constructing the judgment matrix. The eigenvector is the relatively important sorting weight of the index factor of this level for a factor in the upper level. When the judgment matrix constructed by AHP is used, whether the obtained result is reasonable or not requires a one-time inspection of the judgment matrix that is sufficiently early.

(1) $$\begin{array}{c} CI=\frac{\lambda_{\max}-n}{n-1}\text{,} \end{array}$$

where *λ*_max_ is the largest eigenvalue.

Random consistency index *RI* is introduced, and specific values are demonstrated in Table 2.

The consistency ratio is

(2) $$\begin{array}{c} CR=\frac{CI}{RI}\text{,} \end{array}$$

where *RI* is the random consistency index.

Finally, there is a hierarchical total ordering and one-time inspection. It calculates the relative important weights of all index factors to the highest level, that is, the weight vector of index combination. This process is called total ranking of levels. The determination of the weight vector of the realization index combination is conducted from the highest to the lowest level. Like indicator weight vector, the indicator combination weight vector may be tested once.

### 3.2. BP Network and SFLA Algorithm

As the amount of data grows exponentially, so does the complexity of the data. Commonly used simple perceptrons and basic machine learning algorithm rules such as logistic regression can no longer meet the current needs, and machine learning algorithms with more powerful processing capabilities are needed to process data. Compared with the basic learning algorithm, the error back propagation algorithm is more outstanding. The BP algorithm can not only be used in multilayer feedforward neural networks but it can also be used in other types of networks. The structure of BP is demonstrated in Figure 2.

Neurons to each layer are interconnected with neurons in adjacent layers. Data samples pass data into the model through the input layer. After calculation of the hidden layer, information is transmitted to each neuron of the output layer, and this step is called the forward propagation process. When the results output by the output layer of network do not match results of test samples, the neural network model can follow the direction of error reduction. It continuously backpropagates the error from the output layer to the hidden layer and then to the input layer. Weights of neurons in each layer are adjusted accordingly through the back-propagated error signal. After the error goes from back to front, the forward propagation is restarted after a new model is obtained. After repeated execution, the error between the output and the result in the sample is reduced to a predetermined acceptable range, or all iterations are completed. Finally, the final calculation result is returned by the output layer. The forward propagation and backpropagation of BP network are divided into the following steps:

(3) $$\begin{array}{c} y_{i}=f\left(\sum_{i=1}^{N}w_{i}x_{i}+b_{i}\right)\text{,}\\ Loss=\sum_{i=1}^{N}{\left(y_{i}-o_{i}\right)}^{2}\text{,}\\ w^{\prime }=w-∆w^{\prime }\text{,}\\ b=b-∆b, \end{array}$$

where *w* is weight, *b* is bias, and *x* is feature.

The first advantage of the BP network is its capacity to map nonlinearly. An input-to-output mapping function is what the BP neural network accomplishes in essence. A three-layer neural network may accurately model any nonlinear continuous function according to mathematical theory. The BP network's excellent nonlinear mapping capabilities make it ideal for solving problems involving complicated internal systems. The second is the ability to learn and adapt on by themselves. To learn and remember, the BP network uses a learning algorithm that automatically extracts plausible rules from the data and adaptively memorizes these rules in its weights during training. In the third area, the BP network has a good generalization capacity, which allows it to apply learning to new information. Tolerance for error is the fourth quality. Global training results are not affected by the loss of local or partial neurons in the BP network.

However, the BP network also has shortcomings and deficiencies. The first is the problem of local minimization. The BP network is a local search optimization method that addresses a challenging nonlinear problem. Network training will fail if the network weights are gradually shifted in the direction of regional improvement, which will cause the algorithm to veer off course and reach local extremes. BP neural networks, on the other hand, are extremely sensitive to their initial weight. Different weights at the start of the network tend to lead to different local minima. Second, the BP neural network algorithm has a slow convergence rate. A complex objective function must be optimized for the BP neural network algorithm, which is essentially a gradient descent method. As a result, the BP algorithm will be rendered ineffective due to the emergence of the zigzag phenomenon. The third difference is that the BP network structure is different in each case. To choose a BP network structure, there is no uniform and thorough theoretical guidance. It is a skill that, in most cases, can only be acquired by the actual use. Overfitting may occur if the network structure is excessively massive, resulting in worse network performance and poorer fault tolerance. Selecting very few nodes may result in a network that fails to converge.

In view of this shortcoming, this paper decided to use the SFLA to optimize initial weight threshold. SFLA can be described as a randomly generated population of frogs in a pond. All individuals in the population are scattered throughout the swamp, and their ultimate goal is to find the nearest location for food. Each of these frogs also has its own cultural characteristics, and the cultural characteristics of each frog is quite a solution to the problem. The entire frog colony is divided into different subgroups, and each subgroup also has its own specific cultural characteristics. The cultural characteristics of each frog can influence and be influenced by other frogs and will evolve with the evolution of subgroups. When the subgroup evolves to a certain stage, the global information exchange is carried out between each subgroup, and then the subgroup is redivided, and the operation is repeated until the optimal solution is found. All in all, the SFLA algorithm can be understood as a process of the evolution of the cultural characteristics of an individual influencing each other and the global transfer of information between subgroups.

The SFLA algorithm mainly includes two core steps: global search and local search. The global search is initialized first, and the second step is used to simulate a subgroup. For the entire population, there are several frogs in a specific area, and the fitness value of each individual is calculated. The third step is to determine the initial optimal solution, sort the frog individuals in the total group in the ascending order of fitness value, and then record the location of the best frog in the population as the optimal solution. The fourth step is to divide the subgroup, that is, divide the sorted frog group into several subgroups on average. The fifth step is the independent evolution of subgroups, recording the frog with the best fitness and the worst fitness in the subgroup and evolving frog individuals in each subgroup through local search. The sixth step is to judge to stop the iteration when the predetermined number of iterations decreases or at least one individual frog reaches the optimal position. Then it means that the optimal solution has been found, and the iterative optimization can end; otherwise, go back to the previous step to continue optimization. The seventh step is mixed recombination, which recombines all evolved subgroups to form a new group. Then calculate fitness of each individual and then reorder to redivide subgroups so as to continue to iterate to obtain optimal solution.

In the local search process, the first step is to record the best and worst individuals in each subgroup. The second step is to update the worst frog position in the current subgroup through the local optimal solution. The update method is equations (4) and (5). After the update, if the resulting frog is better than the original frog, then replace the original frog with the calculated value. Otherwise, replace the original value with the optimal value, and continue to execute the corresponding formula, if there is still no improvement, a new value is randomly initialized. Then repeat the operation until the number of local iterations is reached, and return to the results in the global search for mixed reorganization and reoperation until the termination condition is met.

(4) $$\begin{array}{c} D=r*\left(X_{b}-X_{w}\right)\text{,} \end{array}$$

(5) $$\begin{array}{c} X_{w}^{\prime }=X_{w}+D\text{,} \end{array}$$

where *r* is a random number, *X*_*b*_ is the best fitness frog, and *X*_*w*_ is the worst fitness frog.

The SFLA algorithm is a combination of advantages based on both the meme algorithm and particle swarm algorithm. The SFLA algorithm has fewer parameters, and the search strategy is also simple and easy to understand and implement. The frog population is grouped based on the average, according to the characteristics of the opposite information, and then a local search is carried out in the subgroup so as to achieve the effect of speeding up the convergence speed. Moreover, SFLA strengthens the information exchange in each subgroup through the mixed reorganization of subgroups, thereby improving the search speed and having strong robustness.

In the local search process of the SFLA algorithm, its step size formula is relatively simple, and it is still unsatisfactory in efficiency to update the worst solution of the subgroup through this single compensation formula. The SFLA algorithm only pays attention to the worst individual in the calculation not only by ignoring the individual differences among frogs in each subgroup but also by ignoring other individuals with poor fitness. It does not pay enough attention to relationship between the global optimal fitness and the local optimal fitness. Therefore, the SFLA algorithm is also prone to the problem of low accuracy. The SFLA algorithm is proposed via the algorithm meme, calculus algorithm, and particle swarm algorithm. Similar to many heuristic search algorithms, the parameter selection of the SFLA algorithm also has no clear theoretical basis.

### 3.3. Improved SFLA and ISFLA-BP Algorithm

This work aims to improve shortcomings for traditional SFLA, and specific measures are used to improve the evolutionary step formula and the individual evolution of frogs. The method of updating the individual step size of frogs in the traditional SFLA algorithm is slightly blind, ignoring the individual differences of the worst frogs in each subgroup. This work proposes an improved evolutionary step (IES) strategy to adaptively adjust the moving step size, making the search of each individual more scientific and reasonable.

(6) $$\begin{array}{c} D=\left\{\begin{array}{c} Ran\;d*\left(X_{b}-X_{w}\right),f_{i}<f_{avg}^{\prime }\text{,}\\ Ran\;d*\left[\lambda \left(X_{g}-X_{w}\right)+\left(1-\lambda \right)\left(X_{w}-X_{g}\right)\right],\\ Ran\;d*\left(X_{w}-X_{g}\right),f_{i}>f_{avg,} \end{array}\right.\;f_{avg}^{\prime }\leq f_{i}\leq f_{avg}\text{,} \end{array}$$

where *λ* is the learning factor.

In addition, this work introduces a mutation operator on the basis of the above formula. The algorithm replaces the random numbers in the step size update formula with the mutation operator and introduces an expression related to the direction of the evolutionary band so as to avoid the worst individual from changing too much of the random number on the basis of improving the convergence speed. This trapping in a local minimum area reduces the convergence accuracy and can further improve the convergence speed.

(7) $$\begin{array}{c} D=\left\{\begin{array}{c} \frac{k_{\max}-k}{k_{\max}}*\left(X_{b}-X_{w}\right),f_{i}<\;f_{avg}^{\prime }\text{,}\\ \frac{k_{\max}-k}{k_{\max}}*\left[\lambda \left(X_{g}-X_{w}\right)+\left(1-\lambda \right)\left(X_{w}-X_{g}\right)\right],\\ \frac{k_{\max}-k}{k_{\max}}*\left(X_{w}-X_{g}\right),f_{i}>f_{avg,} \end{array}\right.f_{avg}^{\prime }\leq f_{i}\leq f_{avg}\text{,} \end{array}$$

where *k*_max_ is the maximum iteration, and *k* is the current iteration

By introducing a mutation operator into the adaptive step size update formula, the influence of being trapped in a local polar cell caused by the uncertainty of random numbers is avoided, and the convergence speed can be further improved on the basis of the adaptive formula.

In addition, this work uses an improved individual evolution (IIE) of frogs. Each selection of the SFLA algorithm in the local search evolves the worst individual in the subgroup, which is updated and then reordered. It cyclically and independently evolves in this way, eventually making the entire subgroup move towards the optimal solution. However, this evolutionary method is not efficient when the population size is too large or the sample dimension is too high. In the improved evolution method, in the process of independent evolution, the frog subgroup is no longer limited to updating the worst frog individuals but selects and updates some individuals with poor fitness. The other steps of the individual evolution method, such as the evolution formula and the global search strategy, do not make any changes. By improving the evolution method, the subgroup can be quickly converged and the solution speed can be improved.

There is a lot of experience with the BP network in terms of both theory and practice. A local optimum can easily be reached since the initial weights and thresholds have been chosen incorrectly, resulting in an inability to get close to the expected value. Swarm intelligence is used in the modified ISFLA algorithm, which is a global search method. A new ISFLA-BP model for small and medium-sized business digital transformation maturity assessment is presented in this study. The initial weight threshold of the BP network is searched globally using the ISFLA algorithm to determine the best initial weight threshold, enhancing convergence and avoiding as much as possible falling into the local optimum. The pipeline of ISFLA-BP is demonstrated in Figure 3.

The ISFLA-BP process used to evaluate the digital transformation maturity of small and medium-sized startups is divided into the following steps. The first step is to obtain the initial BP network model structure as a three-layer network and initialize range for weight thresholds. The second step is to find optimal solution in initialized weight threshold range through the ISFLA algorithm. The third step is to return the optimal solution to BP as the optimal parameter. The fourth step is to perform forward propagation, calculate the actual output value of the data sample, and calculate the sum of squares of the error between the actual value and the expected output. If error sum of squares is less than error precision, then stop training. Otherwise, through backpropagation, update the connection weights and thresholds, perform forward propagation again, and compare the sum of squares of errors until the sum of squares of errors is less than the error precision. The fourth step is to test the network after training.

## 4. Experiment

### 4.1. Determination of the Indicator Weight

This work divides the evaluation indicators of digital transformation maturity into the target layer (A), the criterion layer (B), and the indicator layer (C). The AHP multicriteria method is utilized to calculate weights of the criterion layer B relative to the target layer A. The data are demonstrated in Table 3.

The weights of the indicator layer relative to the criterion layer are determined in Tables 4to 7.

Through the judgment matrix, the single-level ranking of the indicators of each level is obtained, and then the total hierarchical ranking relative to the target layer is obtained according to the single-level ranking. The weight of the indicator layer relative to the target layer is determined in Table 8.

It can be concluded from the table that the weights of the eight indicators C2, C3, C4, C5, C9, C10, C12, and C13 are above 0.05, which are relatively important and have a greater impact on the maturity of digital transformation of small and medium-sized entrepreneurial enterprises.

### 4.2. Evaluation of the ISFLA-BP Algorithm

This work first evaluates the training process of ISFLA-BP, analysis object is the changing trend of the loss during the training process, as demonstrated in Figure 4.

As the training progresses, the loss of the ISFLA-BP network decreases. When training reaches 3000 iterations, network loss stabilizes. After that, ISFLA-BP is compared with other methods, and data are demonstrated in Figure 5.

Compared with other machine learning methods, ISFLA-BP network can achieve the highest accuracy and recall rate for digital transformation maturity assessment of small and medium-sized startups. Compared with other methods, different degrees of performance improvement can be obtained. ISFLA-BP utilizes the improved evolutionary step (IES) strategy to promote SFLA to verify effectiveness for this improved strategy, and this experiment compares the performance of IES and traditional evolutionary step (TES). The comparison data are demonstrated in Figure 6.

Compared with the traditional TES method, after using the IES strategy, the precision and recall rate are increased by 1.3% and 1.4%, respectively, which verifies the superiority of the IES strategy. ISFLA-BP utilizes the improved individual evolution (IIE) strategy to promote SFLA to verify effectiveness for this improved strategy, and this experiment compares the performance of IIE and traditional individual evolution (TIE). The comparison data are demonstrated in Figure 7.

Compared with the traditional TIE method, after using the IIE strategy, the precision and recall rate are increased by 1.1% and 1.3%, respectively, which verifies the superiority of the IIE strategy. To verify the feasibility of using the improved SLFA strategy to optimize BP, performances of traditional BP, SFLA-BP, and ISFLA-BP are compared respectively, and the comparison data are demonstrated in Figure 8.

Compared with the traditional BP network, after using SFLA for optimization, the accuracy and recall rate of the network have increased, and the convergence time has become shorter, which shows that it is feasible to utilize SFLA to optimize the BP network. However, after improving the SFLA algorithm, these indicators can be further improved, which verifies the feasibility of the improvement measures for SFLA. Finally, this work evaluates the impact of different hidden layer nodes on the performance of the ISFLA-BP network, and the comparison data are demonstrated in Figure 9.

After the number of hidden layer nodes is changed, both the precision and recall rates of the ISFLA-BP network change. Its change trend first shows an increase and then a decrease. When the parameter is changed to 5, the highest precision and recall rate can be obtained.

## 5. Conclusion

The nation's economy relies heavily on small and medium-sized businesses. The digital transformation of small and medium-sized entrepreneurial companies is an important road for the country to gain economic power and high-quality economic development in the context of supply-side structural reform. Although a large number of companies have sensed the urgency of digital transformation and have invested significant resources in promoting the integration of digital technologies, only a few companies have achieved significant performance improvements. The digital economy has become an important force to promote the transformation of the national economy from new and old kinetic energy and also provides opportunities for enterprise development to change lanes and overtake. The assessment of enterprises' digital transformation maturity is significant in the digital transformation process. First, this work establishes an evaluation index system for the maturity of digital transformation of small and medium-sized entrepreneurial enterprises, establishes a hierarchical structure for each index via the AHP method in the multicriteria framework, establishes a three-level basic framework, and calculates the weights of evaluation indicators. Second, this work establishes a BP network model for enterprise digital transformation maturity assessment based on AHP and establishes a three-layer BP network. This work aims to optimize BP network using the improved ISFLA algorithm. It improves the adaptive step size update formula in the SFLA algorithm by using the mutation operator and improves the evolution method of the worst individual of the frog to the simultaneous evolution of multiple poor individuals. The constructed ISFLA-BP algorithm is then used to evaluate the digital transformation maturity of small and medium-sized startups. Finally, systematic and comprehensive experiments are carried out to verify the superiority and feasibility of the method.

## Figures and Tables

**Figure 1:** The evaluation index system.

**Figure 2:** BP structure.

**Figure 3:** ISFLA-BP pipeline.

**Figure 4:** Training loss for ISFLA-BP.

**Figure 5:** Comparison of different methods.

**Figure 6:** Comparison of the IES and TES strategy.

**Figure 7:** Comparison of the IIE and TIE strategy.

**Figure 8:** Comparison of different BPs.

**Figure 9:** Evaluation of the hidden node.

**Table 1:** Basic meaning of the scale.

Scale	Meaning
1	Same importance
3	Former is important
5	Former is slightly important
7	Former is obviously important
9	Former is absolutely important
2, 4, 6, 8	Intermediate value of adjacent judgments
1, 1/2,…, 1/9	Ratio of influence is exactly the reciprocal

**Table 2:** RI value.

*n*	1	2	3	4	5	6	7	8	9
*RI*	0	0	0.52	0.89	1.12	1.26	1.36	1.41	1.46

**Table 3:** Judgment matrix of the criterion layer relative to the target layer.

A	B1	B2	B3	B4	Weight
B1	1	0.5	0.5	3	0.19
B2	2	1	0.5	4	0.29
B3	2	2	1	5	0.44
B4	0.33	0.25	0.20	1	0.08

**Table 4:** Judgment matrix of the indicator layer relative to B1.

B1	C1	C2	C3	Weight
C1	1	0.33	0.33	0.14
C2	3	1	1	0.43
C3	3	1	1	0.43

**Table 5:** Judgment matrix of the indicator layer relative to B2.

B2	C4	C5	C6	C7	C8	C9	Weight
C4		0.33	4	4	3	1	0.2
C5	3.	1	5	5	4	3	0.4
C6	0.25	0.2	1	0.5	0.33	0.25	0.05
C7	0.25	0.2	2	1	0.33	0.2	0.06
C8	0.33	0.25	3	3	1	0.33	0.1
C9	1	0.33	4	5	3	1	0.19

**Table 6:** Judgment matrix of the indicator layer relative to B3.

B3	C10	C11	C12	C13	Weight
C10	1	5	3	3	0.54
C11	0.2	1	0.50	0.50	0.1
C12	0.33	2	1	1	0.18
C13	0.33	2	1	1	0.18

**Table 7:** Judgment matrix of the indicator layer relative to B4.

B1	C14	C15	C16	Weight
C14	1	0.17	0.2	0.08
C15	6	1	2	0.58
C16	5	0.50	1	0.34

**Table 8:** Evaluation system weight coefficient.

Indicator	Weight
C1	0.027
C2	0.082
C3	0.082
C4	0.058
C5	0.116
C6	0.015
C7	0.017
C8	0.029
C9	0.056
C10	0.238
C11	0.044
C12	0.079
C13	0.079
C14	0.006
C15	0.046
C16	0.027

## Data Availability

The datasets used during the current study are available from the corresponding author on reasonable request.
